# A Geometric Morphometrics Approach for Sex Estimation Based on the Orbital Region of Human Skulls from Bosnian Population

**DOI:** 10.1155/2023/2223138

**Published:** 2023-04-14

**Authors:** Zurifa Ajanović, Uzeir Ajanović, Lejla Dervišević, Haris Hot, Alma Voljevica, Elvira Talović, Emina Dervišević, Selma Hašimbegović, Aida Sarač-Hadžihalilović

**Affiliations:** ^1^Department of Anatomy, Faculty of Medicine, University of Sarajevo, 71 000 Sarajevo, Bosnia and Herzegovina; ^2^Department of Information Technologies, Faculty of Engineering, Natural and Medical Sciences, International Burch University, 71 000 Sarajevo, Bosnia and Herzegovina; ^3^Department of Forensic Medicine, Faculty of Medicine, University of Sarajevo, 71 000 Sarajevo, Bosnia and Herzegovina; ^4^Department of Ophthalmology, General Hospital Serbia, 71 123 East Sarajevo, Bosnia and Herzegovina

## Abstract

**Background:**

Understanding the anatomy and morphological variability of the orbital region is of great importance in clinical practice, forensic medicine, and biological anthropology. Several methods are used to estimate sex based on the skeleton or parts of the skeleton: classic methods and the geometric morphometric method. The objective of this research was to analyse sex estimation of the orbital region on a sample of skulls from a Bosnian population using the geometric morphometric method.

**Materials and Methods:**

The research was conducted on three-dimensional models of 211 human adult skulls (139 males and 72 females) from the Osteological Collection at the Faculty of Medicine in Sarajevo. The skulls were recorded using a laser scanner to obtain skull 3D models. We marked 12 landmarks on each model to analyse sexual dimorphism. Landmarks were marked using the program Landmark Editor. After marking the landmarks, we used the MorphoJ program to analyse the morphological variability between male and female orbital regions.

**Results:**

After Procrustes superimposition, generating a covariant matrix, and introducing sex as a variable for classification, a discriminant functional analysis (DFA) was applied which determined the estimation for males with 86.33% accuracy and for females with 88.89% based on the form of the orbital region. The results of regression analysis showed that the size of the orbital region has a statistically significant effect on its shape's sexual dimorphism. After excluding the influence of size and providing DFA, we concluded that sex estimation was possible with 82.01% accuracy for males and 80.55% accuracy for females based on the shape of the orbital region in the examined sample.

**Conclusion:**

Sex estimation based on the orbital region was possible with more than 80% accuracy for both sexes, which is a high percentage of correct estimation. Therefore, we recommend using the orbital region of the skull for sex estimation.

## 1. Introduction

Understanding the anatomy and morphological variability of the orbital region is of great importance in clinical practice, forensic medicine, and biological anthropology. The analysis of the morphological variability of the orbital region has found application in the estimation of sex in forensic medicine [1]. Several methods are used to estimate sex based on the skeleton or parts of the skeleton. Classic methods, such as quantitative and qualitative methods, are based on describing the morphological variability between male and female skeletons or measuring defined diameters and comparing them between the sexes [2]. In recent times, methods based on the application of computer programs have been used whose task is to observe even the smallest morphological variability of the examined structures [3].

In the literature is a study where classical morphometry was used for the analysis of sex differences in the orbit [4].

When estimating the sex of skeletal remains, it is important to know the existence of population differences in the skeleton. Created formulas for estimating the sex of one population do not show the same degree of accuracy if they are applied to a sample from another population. These differences are conditioned by hormonal status and differences in climate, food, and culture [5].

Geometric morphometric techniques make it possible to quantify the shape variables of morphological structures. Geometric morphometrics provides an opportunity to analyse the overall shape of a structure, regardless of curvatures and protrusions, using landmarks. Based on the position of the landmarks on the examined structure, using geometric morphometric programs, the existing differences are highlighted, and whether the observed differences are statistically significant has been examined, which is impossible using classic methods [6].

The geometric morphometric method differs from classical morphometrics in that the definition of the shape of morphological characteristics of objects coincides with the mathematical definition of the shape. Shape is defined as a set of geometric information that is immutable with respect to scaling, translation, and rotation [7].

The geometric morphometric method was used to study sexual dimorphism not only of the skull but also of other parts of the skeletal system, and in the literature, we can find studies which analysed sexual dimorphism of long bones such as long bones of the upper extremity [8], scapula [9], clavicle [10], pelvic bones [11], long bones of the lower extremity [12], and spine [13].

The geometric morphometric method is widely used in tracking changes in the shape and size of the skeletal system, including the skull as part of that system, during evolutionary development [14].

Authors around the world use the geometric morphometric method to investigate shape difference between examined groups in different populations and in different scientific fields [15–19].

The geometric morphometric method has found its application in many branches of medicine. It offers solutions in the reconstruction of missing parts of the skeletal system [20].

Then, the geometric morphometric method has found its application in the fashion industry, as for example, Valenzano and the authors in their research use geometric morphometrics to investigate the attractiveness of the face in the examined women [21].

Also, in the literature, there are studies that use classic methods and the geometric morphometric method in their investigations of sexual dimorphism in order to examine the accuracy of the results obtained using the geometric morphometric method, where they concluded that the geometric morphometric method is as reliable as classical morphometrics.

Ross's study investigated whether there were differences in the results of sex estimation using different methods. The author concluded that the results of skull classification (black or white population) using morphometrics were comparable to the results obtained using discriminant analysis [22].

In 2016, Toneva and fellow authors compared the research results obtained using classical morphometrics with the results obtained using digital technologies on three-dimensional models of the same sample, and the research results were similar regardless of the method used [23].

The importance of the geometric morphometric method in science, its development, progress, and instructions for its use in further research have been presented by a number of authors [24–27].

In 2002, Richtsmeier et al. also cited the benefits of the geometric morphometric method in investigations of sexual differences [28], both in anthropology and in other fields of biological research, and used it in animal [29, 30] and plant research [31].

In his 2018 paper, Klingenberg states that the use of geometric morphometrics in the study of differences in biological structures is incompletely examined and that, in addition to the study of differences in allometry, ontogeny, and sex differences, geometric morphometrics offers solutions in the study of biological systems and other fields [32].

To the best of our knowledge, this method has not been used to analyse sexual dimorphism in the orbital region.

The objective of the research was to analyse sex estimation of the orbital region on a sample of skulls from the Bosnian population using the geometric morphometric method.

## 2. Material and Methods

### 2.1. Sample

Investigation was provided on three-dimensional models of a total of 211 human adult skulls (139 males and 72 females) from the Osteological Collection at the Faculty of Medicine in Sarajevo, after obtaining the approval of the Ethics Committee of the Faculty of Medicine (Number 02-3-4-2377/18). In order to obtain three-dimensional models of the skulls, the skulls of the tested sample were recorded using a laser scanner (Structured Light Scanner SLS-2 by DAVID, Germany). The DAVID Vision system is a mobile system for scanning objects of different geometries with resolution accuracy of 0.05%. The DAVID system (Figure 1) has a calibration plate, stand, projector, camera, and software. After the adjustment and calibration procedures, the skull was then rotated to record a certain number of scans, which are sufficient to make a three-dimensional model of the skull, and can be used in various formats. The projector and camera were mounted on a tripod, and both can be slid along the tripod.

After setting up and calibrating the scanner according to the manufacturer's instructions, three-dimensional models of skulls were recorded. The skull was placed on a rotating stand, and the number of scans (total of 15) was set on a computer connected to the scanner.

The obtained scans were cleaned of artifacts, and everything was removed from the recording except the skull scan itself. After the fusion of the scans, a three-dimensional model was obtained. After obtaining three-dimensional models of all skulls of the examined sample, the models for each skull were saved in .ply file format (Figure 2).

For the analysis of the sex differences of the orbital region, we used 12 landmarks (6 paired anthropometric points): orbitale, maxillofrontal, ectoconchion, supraconchion, subconchion, and frontomalare orbitale which are presented in Table 1 [33].

Table 1 shows landmarks which are used for the analysis of sex differences in the orbital region.

For marking landmarks (Figure 3), we used the program Landmark Editor [34].

### 2.2. Statistical Analysis

Sex estimation of the orbital region of the examined skulls was performed using tests from the MorphoJ program [26]. The total variability on the orbital region of skulls was explored using principal component analysis. In geometric morphometrics, the size of the structure was labelled as the centroid size (CS). Regression analysis was used to analyse the effect of the orbital region size on its shape. Discriminant functional analysis was used to compare sex dimorphism of the orbital region. The level of statistical significance used in the study was *p* = 0.01.

## 3. Results

The analysis of the PC showed that PC1 and PC2 described 37.5% of the total variability of the orbital region taking into account both the shape and size of the orbital region (Figure 4 and Table 2).

Figure 5 shows a clear separation in the form of the orbital region between males and females.

A correct classification test analyses the mean values of these two groups in the form of Procrustean distances or Mahalanobis distances.

The calculated Procrustean distance is 0.0267 and the *p* value was less than 0.001, which showed a significant sex dimorphism in form of the orbital region.

Results of DFA showed that accuracy for sex estimation for males was 86.33% and 88.89% for females (Table 3).

Figure 6 shows the results of the DFA of sex differences in the form of the orbital region of the examined skulls.

Regression analysis examined a significant effect of the size of the orbital region on its shape. The *p* value for regression analysis results was less than 0.001 (Figure 7).

PC1 and PC2 analysis of the orbital region shape described 36.443% of the total variability in the shape of the orbital region (Table 4 and Figure 8).

Results of DFA showed that accuracy for sex estimation of males using the shape of the orbital region was 82.01% and 80.55% for females (Table 5 and Figure 9).

The interval of orbital shape changes is shown in Figure 10 as a wireframe.

## 4. Discussion

Geometric morphometric analysis of the shape and size of bones is a relatively young, but very interesting, method for sex estimation. In our research, geometric morphometrics was applied for sex estimation based on the orbital region of human skulls. Results showed that sex estimation was possible with 86.33% accuracy for males and 88.89% accuracy for females based on the shape and size of the orbital region. Results of the effect of the size of the orbital region on its shape showed a statistically significant effect. When we excluded the effect of the size and analyse sex estimation based on the shape of the orbital region, results showed that sex estimation was possible with 82.01% accuracy for males and 80.55% accuracy for females.

The percentage of correct estimation based on the orbital region was about 80% accuracy for both sexes in the sample from the Bosnian population.

We compared our results with the results of authors whose studies were conducted on samples from different populations and with the application of different methodologies.

On a sample of 171 skulls of known sex from the Greek population, sex estimation based on the shape of the orbital region was possible with 74.4% accuracy for males and 70.4% accuracy for females, while based on the form of the orbital region (size and shape), sex estimation is possible with 83.3% accuracy for males and 82.7% accuracy for females [35].

Previous studies of sexual dimorphism on skulls of American whites showed 87.5% accuracy using the classic methodology which is in agreement with our results [18].

In the study conducted by Bigoni et al. [33] on a sample of 133 human skulls of known sex from Central Europe, sex estimation based on the orbital region was possible with 74% accuracy.

The results of the research by Graillon et al. which was done on 3D reconstructed models, where sex differences in the volume of the orbital cavity were analysed, showed that the volume of the orbital cavity is statistically significantly higher in male skulls than in female skulls. Based on the volume of the orbital cavity, sex estimation was possible with 77.3% accuracy [36].

In the research done by Bassil-Nassif et al. [37], an analysis of the dimorphism between the sexes in the volume of the facial cavities, including the orbital cavity, was also performed. The research results showed that the volume of the cranial cavity was significantly higher in male skulls than in female skulls, but the ratio of the volume of cranial cavities did not show significant differences between sexes [37].

Regensburg et al. [38] examined the accuracy of a new CT scan-based method for estimating orbital cavity volume. The research was repeated by two researchers using the same methodology on the same sample. The precision of the calculations between the two researchers varied from +0.7% to -0.7% for the volume of the orbital cavity. They came to the conclusion that this technique was reliable and precise [38].

Kimmerle et al. [39] conducted a study on 118 skulls of American whites and blacks of known sex, where they tracked 16 anthropometric points on three-dimensional models obtained using a special Microscribe-3DX digitizer and special Morphologika software. They came to the conclusion that the appearance of the skull was influenced by sex, regardless of race, while skulls of different sizes of the same sex do not differ in morphological characteristics [39].

The use of bony landmarks, as in our study, has the possibility of being used on bone material after death but also on living individuals using the technique to visualize the bone system. To estimate sex based on the orbit, some authors used the orbital index calculation. A significantly higher orbital index in females than in males was found in the study of Ezeuko et al. [40] and Ebeye and Otikpo [41] which was in contrast with the findings of Mekala et al. [42]. According to the study of Kaplanoglu et al. [43], orbital diameters were larger in men than in women.

A large number of studies on orbital sexual dimorphism demonstrated its importance for sex estimation and analysis of differences between populations. In the research provided by Husmann and Samson [44], an assessment of the practical importance of these assessments was investigated. The diameters of the orbital cavity were measured, the orbital index was calculated, and the differences between the male and female sexes of blacks and whites from the Hamann-Todd collection were assessed. The authors also examined the repeatability of these measurements. Geometric morphometrics was applied to examine the shape differences of the orbital border. The research results showed that there are significant differences in the index and in the geometric morphometric study. The differences between measurements by two different researchers were small.

Brown and Maeda explored the differences between orbital cavities of the recent East Asian population and their ancestors. They came to the conclusion that in the course of evolution, there was a decrease in the size and robustness of the orofacial skeleton, including the orbit [45].

In a study conducted on a sample of Bantu South Africans, Pretorius et al. [46] used geometric morphometrics to analyse sexual dimorphism of the incisura ischiadica major, angulus mandibulae, and orbita. The largest sexual dimorphism was observed on the incisura ischiadica major, as expected. The orbit had more pronounced sexual dimorphism than the angulus mandibulae.

By using CT scans, Andrades et al. [47] found that the average orbital volume in men is bigger than that in women and age group analysis demonstrated a slow increase in orbital volume beyond 30 years (*p* = 0.98). Age differences were not considered in our study. Previous research has shown that the diameters of the orbital cavities are larger in men. The width and height of the orbital cavities decreased during life, while the depth of the orbital cavity increased. The increase in the depth of the orbital cavities was more pronounced in women [48–50].

The results of our research showed that the existing morphological differences of the orbital region are conditioned by sex variations without taking into account the age of the examined skulls.

The results of studies conducted on a sample of skulls from the Bosnian population showed the existence of sex differences on different parts of the skull with the application of different methodologies [51–58].

The results of this study contribute to the formation of specific models for sex determination of the Bosnian population.

## 5. Conclusion

Geometric morphometrics showed that there is statistically significant sexual dimorphism in the orbital region of the examined skulls. Sex estimation based on the orbital region was possible with more than 80% accuracy for both sexes, which is a high percentage of correct estimation. Therefore, we recommend using the orbital region of the skull for sex estimation.

## Figures and Tables

**Figure 1:** HP 3D Structured Light Scanner Pro S2 Laser Scanner (DAVID SLS-2); camera, projector, and stand (b); calibration plate and rotating stand (a).

**Figure 2:** Assembling the scans and obtaining a three-dimensional model.

**Figure 3:** Designation of specific points in the Landmark Editor program for the orbital region.

**Figure 4:** Principal component analysis of change in the form of the orbital region on examined skulls. Blue circles represent the mean values of landmarks; blue lines represent the direction and intensity of changes in the mean values of landmarks on the examined sample.

**Figure 5:** Morphospace of the first two principal components of the form variation in the orbital region of examined skulls between sexes (males (M) are indicated by the blue colour, females (Ž) by the pink colour).

**Figure 6:** Discriminant functional analysis of sex differences in the form of the orbital region of the examined skulls. Males (M) are represented by blue histograms, females (Ž) by pink histograms.

**Figure 7:** Regression of size (expressed as centroid size) on the shape of the orbital region. The analysis demonstrated statistically significant influence. M: male; Ž: female (*p* < 0.001 with 10,000 repetitions).

**Figure 8:** Morphospace of the first two principal components of the shape variation in the orbital region of the examined skulls between sexes (male are indicated by blue colour (M, male), females by pink colour (Ž, female)).

**Figure 9:** Discriminant functional analysis of sex differences in the shape of the orbital region of the examined skulls. Males (M) are represented by blue histograms, females (Ž) by pink histograms.

**Figure 10:** Wireframe of sex differences in the orbital region of the examined skulls.

**Table 1:** Landmarks used for analysis of sex differences in the orbital region of the examined skulls.

Landmarks	Position
Orbitale	Most inferior point on the inferior margin of the orbit
Maxillofrontale (mf)	Intersection of the frontomaxillar suture and medial margin of the orbit
Ectoconchion (ek)	Intersection of the lateral margin of the orbit and the line from the mf parallel with the superior margin of the orbit
Supraconchion	Intersection of the superior margin of the orbit and normal to the line mf-ek
Subconchion	Intersection of the inferior margin of the orbit and normal to the line mf-ek
Frontomalare orbitale	Intersection of the frontozygomatic suture and the lateral margin of the orbit

**Table 2:** Eigenvalues and percentage of orbital region form variability described by principal component analysis (PCA).

PC axis	Eigenvalues	Percentage of variability (%)	Cumulative percentage of variability (%)
1.	0.00059290	21.810	21.810
2.	0.00042667	15.696	37.506
3.	0.00038130	14.027	51.532
4.	0.00029747	10.943	62.475
5.	0.00026672	9.812	72.287
6.	0.00022464	8.264	80.550
7.	0.00019161	7.048	87.599
8.	0.00011938	4.391	91.990
9.	0.00007778	2.861	94.851
10.	0.00005824	2.142	96.994

**Table 3:** Sex estimation based on the form of the orbital region of the skulls.

	Sex estimation		Total
Sex			
Male	120	19	139
Female	8	64	72
Total	128	83	211

**Table 4:** Eigenvalues and percentage of orbital region shape variability between sexes described using principal components analysis (PCA).

PC axis	Eigenvalues	Percentage of variability (%)	Cumulative percentage of variability (%)
1.	0.00056083	21.654	21.654
2.	0.00038302	14.789	36.443
3.	0.00036229	13.988	50.431
4.	0.00028556	11.026	61.457
5.	0.00026669	10.297	71.754
6.	0.00022462	8.673	80.427
7.	0.00017479	6.749	87.176
8.	0.00011936	4.609	91.784
9.	0.00007616	2.941	94.725
10.	0.00005563	2.148	96.873

**Table 5:** Test of correct classification between sexes based on the shape of the orbital region of the examined skull.

	Sex estimation		Total
Sex			
Male	114	25	139
Female	14	58	72
Total	128	83	211

## Data Availability

The data used in this study are available from the corresponding author upon request.
